# Erythrocytic, Enzymatic, and Histological Markers of Oxidative Stress in Subacute and Chronic Stage Infections in Wistar Rats (*Rattus norvegicus*) Infected with *Trypanosoma brucei brucei*

**DOI:** 10.1155/2023/3590893

**Published:** 2023-04-17

**Authors:** Z. Abubakar, N. T. Dabo

**Affiliations:** ^1^Department of Biological Sciences, Faculty of Science, Federal University Dutse, Jigawa, Nigeria; ^2^Department of Biological Sciences, Faculty of Life Science, College of Natural and Phamaceutical Sciences, Bayero University, Kano, Nigeria

## Abstract

Trypanosomiasis is a complex of diseases caused by a haemoprotozoan parasite of medical and veterinary importance. One of the leading factors that cause morbidity and death in trypanosomiasis is oxidative stress. The oxidative stress biomarkers in trypanosomiasis at the subacute and chronic stages of infection were investigated in this study. A total of twenty-four Wistar rats were used; the animals were placed in two groups: group A (subacute and chronic) and group B (control). The weight and body temperature of the experimental animals were determined using a digital weighing balance and thermometer. A hematology analyzer was used to determine the erythrocyte indices. Spectrophotometry was used to estimate enzyme (superoxide dismutase, catalase, and glutathione) activities in the serum, kidney, and liver of experimental animals. Liver, kidney, and spleen were harvested and analyzed for histological changes. The mean body weight of the infected decreased compared to the control (*P* < 0.05). The mean body temperature of infected individuals increased (35–37°C) compared to the control (*P* < 0.05). The erythrocyte indices of the infected and control groups indicate a significant decrease (*P* < 0.05). In erythrocyte indices, only MCHC indicated a nonsignificant decrease (*P* > 0.05). The SOD of serum shows a significant increase (*P* < 0.05), and no significant increase SOD (*P* > 0.05) in kidney and the liver SOD indicates a significant decrease (*P* < 0.05). The serum, kidney, and liver show a significant increase (*P* < 0.05) in CAT. The serum GSH from the findings indicates a nonsignificant increase (*P* > 0.05), and the kidney and liver GSH shows a significant increase (*P* < 0.05). The correlation analysis for SOD shows nonsignificant negative correlation for serum/kidney, and the serum/liver and kidney/liver show significant positive correlation. The result of CAT shows significant correlations for serum and kidney, serum and liver, and kidney/liver with a positive correlation. The GSH result shows no significant negative correlation for serum/kidney and no significant positive correlation for serum/liver and kidney/liver. The histological damage in the kidney, liver, and spleen was much higher in the chronic stage than in the subacute stage and no tissue damage in the control group. In conclusion, subacute and chronic stage trypanosome infection is associated with changes in hematological indices, antioxidants of the liver, spleen and kidney, and histological architecture.

## 1. Introduction

Trypanosomiasis is a complex of diseases caused by a haemoprotozoan flagellated parasite of the family Trypanosomatidae and genus Trypanosoma, with different species of human and veterinary importance [1]. Oxidative stress is an imbalance between radical-generating (oxidants) and radical-scavenging (antioxidants) activity, resulting in oxidation of products and subsequent damage to tissue and organs [2]. Oxidants are derivatives of molecular oxygen, e.g., O, H2O2, OH (reactive oxygen species, ROS) or NO, and NO2 (reactive nitrogen species, ROS). The notable enzymatic antioxidants include superoxide dismutase (SOD), catalase (CAT), glutathione reductase (GSH), and glutathione peroxidase (GPx) [3].

Evidence has shown that oxidative stress affects the spermatozoa and leads to a number of reproductive diseases such as pregnancy complications (spontaneous abortion, recurrent pregnancy loss, etc.), infertility, and endometriosis in women [4, 5]. The diagnosis of trypanosomiasis remains a challenge, especially in determining the stage of the disease. Oxidative stress has been identified as playing a key role in the pathological reaction resulting in damage to cells and tissues. Many studies on oxidative stress biomarkers in trypanosomiasis place emphasis on the level of damage caused by oxidative stress; few, if any, have used antioxidant enzymes of different tissues to give a baseline for indicating the sub-acute or chronic stage of the disease. Trypanosomes have two stages: subacute (hemolymphatic) and chronic (meningoencephalitic) in the host. There is a need to categorically differentiate between the two stages of trypanosomiasis in order to give a proper prescription for the treatment of the disease. Oxidative stress biomarkers in different tissues can continuously be explored as a potential strategy to overcome difficulties associated with the diagnosis of trypanosomiasis.

Oxidative stress and toxins from the parasite result in leucopenia, anemia, thrombocytopenia, tissue inflammation and damage, splenomegaly, and cachexia [6]. In recent years, there has been an increasing interest in the field of parasite diagnosis. It is an established fact that infections due to trypanosomes lead to reduced production, infertility, abortion, and death [7].

Oxidation of products and tissue damage in camels as an experimental model has been adopted by many researchers. In a study by Saleh et al. [8], an increase in erythrocytic catalase with a reduction in reduced glutathione and superoxide dismutase was observed in infected *Trypanosoma evansi* camels. The erythrocyte indices show a decrease in infected *Trypanosoma evansi* [8, 9]. Significant reductions in serum catalase, superoxide dismutase, and reduced glutathione have been observed in experimental horses infected with *T. evansi* ([10]; Rashmi et al., 2017). In *T. brucei* infected rabbits, reduction in liver and kidney superoxide dismutase and catalase was observed [11]. In a study of the antioxidant status of *T. evansi* in rats by Omer et al. [12], results indicated that infection in all rats resulted in a fulminating parasitemia. Reduction in erythrocyte parameters of *T. evansi*-control and infected rats indicates macrocytic hypochromic anemia and anisocytosis reduction in the activity of superoxide dismutase in the blood of infected rats. Results obtained indicated that trypanosomiasis caused oxidative stress and induced antioxidant enzymes [12]. Superoxide dismutase deficiency exacerbates the mitochondrial reactive oxygen species and oxidative damage in Chagas disease, and MnSOD deficiency exacerbates the loss in mitochondrial function and oxidative phosphorylation capacity and enhances the myocardial oxidative damage in chagasic cardiomyopathy [13]. Mitochondria-targeted small molecule mitigators of MnSOD deficiency will offer potential benefits in averting mitochondrial dysfunction and chronic oxidative stress in Chagas disease [13]. Increases in the antioxidant enzyme parameter in the blood of *T*. *brucei-*infected rats, a significant reduction in liver SOD, an increase in kidney SOD, an increase in both liver CAT and kidney, and an increase in both liver GSH and kidney GSH [14, 15] were also reported. Oxidative stress is one of the primary events in the pathogenesis of trypanosomiasis. Balogun et al. [16] reported distortion in the observed organs (spleen, kidney, cerebellum, and liver). Infection with *T. brucei brucei* causes oedema, hyperplasia, splenomegaly, tissue necrosis, and inflammation of organs. Trypanosomiasis can also lead to subcutaneous swellings caused by the accumulation of tissue (oedema). This causes an increase in the permeability of blood capillaries and leakage of blood plasma, thereby causing swellings [17]. Interaction between the host immune system and the parasite results in leucopenia, anemia, thrombocytopenia, tissue inflammation and damage (due to oxidative stress and toxins from the parasite), splenomegaly, and cachexia [6]. Red blood cells' damage due to peroxidative damage and destruction by immune cells caused by the parasite directly increase the pathogenesis of the anemia it causes [17, 18]. Oxidative stress is one of the primary events in the pathogenesis of trypanosomiasis [16]; this is because the RBC of the host has reduced antioxidant ability [17]. Studies have shown that a decrease in body temperature, a decrease in body weight, and even death in the absence of drug intervention are key signs of disease morbidity ([16, 19]; and [20]). Infection with trypanosomes is generally known to be associated with an increase in body temperature, which is a result of contact between the parasite and the host's defense system and a decrease in weight due to a loss of appetite on the host's part [17].

## 2. Materials and Methods

### 2.1. Test Organisms

*Trypanosoma brucei brucei* was obtained from the Department of Vector and Parasitology, Nigerian Institute for Trypanosomiasis Research, Kaduna State (NITR) via the Kano State Liaison Office. The parasite was passage onto donor a rat from liquid nitrogen. To obtain the active form, blood obtained from the donor rats by heart puncture was dissolved in phosphate buffer saline, which serves as a medium for passage onto two new Wistar rats. The same was repeated until the parasites' active form was seen microscopically.

### 2.2. Experimental Animals

Thirty healthy adult Wistar rats (*Rattus norvegicus*) were used for the experiment. Composed of fifteen males and fifteen females, weighing 160–240 g (five months old), the animals were purchased from the Department of Biological Sciences, Bayero University, Kano. The experimental animals were acclimatized for 30 days in cages at the laboratory; they were handled in accordance with the guidance of Animal Research Report of *in vivo* Experiment [21].

### 2.3. Sample Size

The animal sample size was determined using the method outlined by Charan and Kantharia [22], “the law of diminishing returns”:

(1) $$\begin{array}{c} E=\text{Total number of animals}–\text{Total number of groups}, \end{array}$$

where *E* is the degree of freedom of analysis of variance.

(2) $$\begin{array}{c} E=\left(7\times 4\right)-4,\\ E=24. \end{array}$$

Therefore, the sample size is 24 animals.

### 2.4. Experimental Design and Parasite Inoculation

Twenty-four animals were randomly placed into two groups (A and B; 12 animals per group). Group A infected group with 12 animals (subacute stage and infected chronic stage) and group B uninfected group with 12 animals (control). The groups were then divided into six subgroups: A1 (subacute stage infection) and A2 (chronic stage infection) six animals per group and B1 (control for A1) and B2 (control for A2) six animals per group following randomization during sacrifice at the subacute and chronic phases of the experiment. Animals in subgroup A were inoculated intraperitoneally with 10^3^ trypanosomes from the infected blood of a donor rat (day 1), with phosphate-buffered saline as a physiological solution to aid infection. Animals in subgroup B received the same phosphate buffered saline without parasites and underwent similar procedures as their counterparts.

### 2.5. Daily Monitoring of Parasitemia, Temperature, and Weight

Using the Herbert and Lumsden [23] method of rapid matching for estimating the host's parasitemia, the parasitemia of the infected groups was monitored on daily basis at 9 am, by preparing a wet mount as described by Dabo and Maigari [7], using the peripheral blood from the tail of the Rat. A drop of blood was placed on a clean glass slide, covered with a cover slip. Each slide was prepared separately and observed under the x40 objective lens of a binocular microscope. The average of parasitemia in 10 fields was used for evaluation of the degree of parasitemia. The rectal temperature was measured at 9 a.m. daily using a digital thermometer. The record was carried immediately after the thermometer made a beep sound, indicating the conclusiveness of the reading. The weight of each animal in an individual group was measured using a weighing balance. Weight was also determined at 9 a.m. on a daily basis.

### 2.6. Sample Collection and Handling

Blood, liver, kidney, and spleen samples from groups A and B were collected at the onset of the parasitemia (first phase of experiment), after randomization from individual group to choose six Wistar rats each group for subacute stage of infection and its control. The Wistar rats were anesthetized, using kitamine injection before samples were collected. The blood samples were collected by heart puncture using a 1 mL syringe and transferred into plain EDTA containers. The organs were identified, removed, and raised with distilled water. For histopathology, organs were preserved in 10% formalin, while for antioxidant enzyme analysis, organs were preserved on ice before being taken to the laboratory for analysis. At the end of the second phase of the experiment, the remaining Wistar rats in subgroups A and B were treated in the same manner as the Wistar rats in the first phase with respect to sample collection and handling.

### 2.7. Analysis for RBC Indices

The RBC index analysis was carried out using an auto analyzer (model number: BK-5000P).

### 2.8. Antioxidant Analysis and Histopathology

For antioxidant markers, analysis was conducted for catalase, superoxide dismutase, and reduced glutathione in the serum, liver, and kidney. Using the catalase assay kit of the solar bio (life science) company (catalogue number BC0200), the superoxide dismutase (SOD) assay kit of the solar bio (life science) company (catalogue number BC0170), and the reduced glutathione of the Elabscience company, a spectrophotometer with model number 721 was used to carry out spectrophotometric analysis. The tissues were processed as described by Barker and Silverton [24].

### 2.9. Data Analysis

All data obtained were analyzed using SPSS Version 23. A one-way analysis of variance was used to determine the significant difference between the means. Post hoc test analysis was done using the Bonferroni multiple comparison test. *P* values less than 0.05 were considered statistically significant. A two-tailed correlation analysis was used to determine the strength of the association with respect to the level of antioxidants in serum, kidney, and liver.

## 3. Results

### 3.1. Mean Body Weight of Experimental Wistar Rats Infected with T. brucei brucei under Subacute and Chronic Stages

The result of the body weight (Figure 1) in the figure shows the mean body weight of the infected groups and control groups and compares weight loss or gain. From the chart, days 1–3 show differences in weight for each individual group while maintaining a static mean body weight. There was an increase in mean body weight in the subacute stage of infection in day 4, and a slight increase was also seen in the chronic stage group and the control subacute stage group. In days 5 and 6, there was no changes in the body weight. A clear trend of decreasing mean body weight in the chronic stage was recorded, while a slight increase in mean body weight in the control chronic stage was seen from days 7 to 11. The mean body weight of the infected rats decreased compared to the control (*P* value ≤ 0.05).

### 3.2. Mean Body Temperature of Experimental Wistar Rats Infected with T. brucei brucei under Subacute and Chronic Stages

The mean body temperature of the infected and control groups (Figure 2) shows a stationary temperature for control sub-acute stage and control chronic stage, while the subacute stage and chronic stage groups show a decrease in temperature (34°C) from day 1 to day 2, respectively, after which the temperature rose in day 3 to 37°C. The temperature of the two control groups maintained 35–36°C throughout the experiment, and only that of the chronic stage control shows a decrease of 34°C was observed in day 9. For the subacute stage, it maintains a temperature of 36°C up to day 6 after a decrease on day 4. The chronic stage group shows stability in temperature at days 5 and 6, followed by a decline at day 7. From day 7, elevations in temperature were seen up to day 9 where it became stable at the highest peak of 37°C. On day 11, a decrease in temperature of 29°C was recorded. The mean body temperature of infected individuals increased (34–37°C) compared to the control (*P* value ≤ 0.05).

### 3.3. Mean Parasitemia of Experimental Wistar Rats Infected with T. brucei brucei under Subacute and Chronic Stages

There was a clear stationary of parasitemia from days 1 to 3 (Figure 3) in both chronic and subacute groups, in days 4 and 5, a rise in parasitemia was observed in both groups. In chronic stage group, the parasitemia kept increasing until at the final day (11) where it raised to a peak of over 800.

### 3.4. Percentage Survival of Experimental Wistar Rats Infected with T. brucei brucei under Subacute and Chronic Stages

The subacute stage group has a 100% survival up to day 6. The chronic stage group has 100% survival up to day 10 and 80% survival day 11 (Figure 4).

### 3.5. Erythrocytic Indices of Experimental Wistar Rats Infected with T. brucei brucei under Subacute and Chronic Stages

Results for erythrocytic indices of trypanosome infected and control groups are presented in the table (Table 1). The PCV of the experimental animals shows the values for subacute stage (27.87 ± 2.21^ab^), subacute stage control (34.72 ± 0.54^ad^), chronic stage (20.46 ± 1.36^bdf^), and chronic stage control (32.57 ± 1.81^f^), with a *P* value (<0.001). The chronic stage is significantly different among the three groups, and a mean difference appears between subacute stage and subacute stage control. The result for Hgb shows *P* value (<0.001), and Hgb values for subacute stage (9.28 ± 0.74^ab^), subacute stage control (11.58 ± 0.18^ad^), chronic stage (6.82 ± 0.45^bdf^), and chronic stage control (10.87 ± 0.60^f^). The chronic stage is significantly different among the three groups, and a mean difference appears between subacute stage and subacute stage control. The table results for MCHC indicate a nonsignificant difference (*P* value = 0.747) in MCHC of subacute stage (33.31 ± 0.05), subacute stage control (33.31 ± 0.06), chronic stage (33.30 ± 0.03), and chronic stage control (33.37 ± 0.03). For MCV, a significant difference (*P* value ≤ 0.001) in MCV of subacute stage (61.44 ± 2.09^b^), subacute stage control (67.86 ± 0.33^d^), chronic stage (53.80 ± 1.56^bdf^), and chronic stage control (66.41 ± 1.92^f^). The mean of chronic stage group is significantly different with the mean of three groups. The table result for MCH indicates a significant decrease (*P* value ≤ 0.001) in MCH at the subacute stage (20.47 ± 0.69^b^), subacute stage control (22.64 ± 0.12^d^), chronic stage (17.92 ± 0.51^bdf^), and chronic stage control (22.16 ± 0.64^f^). The mean of chronic stage group is significantly different with the mean of three groups. The result for RBC from the table shows a significant difference (*P* value ≤ 0.001) in RBC of subacute stage (4.50 ± 0.21^b^), subacute stage control (5.12 ± 0.09^d^), chronic stage (3.78 ± 0.14^bdf^), and chronic stage control (4.88 ± 0.15^f^). The mean of chronic stage group is significantly different with the mean of three groups. The erythrocyte indices of the infected and control groups indicate a significant decrease (*P*value ≤ 0.000) in erythrocyte indices, and only MCHC indicated a nonsignificant decrease (*P*value = 0.747).

### 3.6. Superoxide Dismutase of Experimental Wistar Rats Infected with T. brucei brucei under Subacute and Chronic Stages

The serum SOD from the table (Table 2) shows a *P* value of (0.03) with a mean value for subacute stage (6.24 ± 0.60), chronic stage (7.69 ± 0.80), subacute stage control (5.21 ± 0.97), and chronic stage control (4.70 ± 0.44). From the table, the result of kidney SOD shows a mean value for subacute stage (6.63 ± 1.43), subacute stage control (5.97 ± 1.65), chronic stage (11.06 ± 2.57), and chronic stage control (6.02 ± 1.98) with *P* value (0.23). The means of liver SOD for subacute stage (2.67 ± 0.14^ab^), subacute stage control (4.22 ± 0.44^ad^), chronic stage (0.06 ± 0.00^bdf^), and chronic stage control (3.18 ± 0.42^f^) with *P* value (<0.001). The mean of the chronic stage is different from the means of the three groups, and differences lie between the means of the subacute stage and the subacute stage control.

### 3.7. Catalase Activity of Experimental Wistar Rats Infected with T. brucei brucei under Subacute and Chronic Stages

The serum CAT as provided from the table (Table 3) shows a *P* value (0.011) and mean value for subacute stage (1.58 ± 3.03), subacute stage control (0.97 ± 0.13^d^), chronic stage (1.90 ± 0.24^df^), and chronic stage control (0.98 ± 0.09^f^). Kidney CAT shows mean value for subacute stage (13.67 ± 0.68), subacute stage control (7.11 ± 3.55), chronic stage (15.33 ± 0.56^d^), and chronic stage control (8.43 ± 1.00) with *P* value (0.016). Liver CAT shows a *P* value (0.008) with mean value for subacute stage (2.56 ± 0.21^a^), subacute stage control (2.08 ± 0.18^ad^), chronic stage (3.16 ± 0.19^df^), and chronic stage control (2.08 ± 0.24^f^). Significant difference was seen between chronic stage and subacute stage together with chronic stage and chronic stage control and also between subacute stage and subacute stage control.

### 3.8. Reduced Glutathione of Experimental Wistar Rats Infected with T. brucei brucei under Subacute and Chronic Stages

The result of serum GSH as presented in the table (Table 4) shows a *P* value (0.605) with mean value for subacute stage (0.19 ± 0.032), subacute stage control (0.27 ± 0.128), chronic stage (0.13 ± 0.001), and chronic stage control (0.27 ± 0.109). The kidney GSH shows mean value for subacute stage (0.70 ± 0.067^a^), subacute stage control (1.02 ± 0.065^ac^), chronic stage (0.43 ± 0.061^c^), and chronic stage control (0.78 ± 0.156) with *P* value (0.003). From the table, liver GSH shows a *P* value (0.003), with mean value for subacute stage (0.55 ± 0.117^a^), subacute stage control (0.95 ± 0.076^ac^), chronic stage (0.37 ± 0.050^c^), and chronic stage control (0.72 ± 0.130).

### 3.9. Correlation for Superoxide Dismutase of Infected and Control Groups

The result of correlation analysis from the table (Table 5) for superoxide dismutase shows nonsignificant difference (*P* = 0.517) in correlation for serum and kidney with a positive correlation (0.139), no significant different (*P* = 0.098) for serum and liver with negative correlation (-0.34), and finally another nonsignificant different (*P* = 0.332) for kidney and liver with positive correlation (-0.207).

### 3.10. Correlation for Catalase of Infected and Control Groups

The table (Table 6) shows a correlation analysis for catalase. The result shows significant difference (*P* = 0.044) in correlation for serum and kidney with a positive correlation (0.415), no significant different (*P* = 0.065) for serum and liver with positive correlation (0.383), and significant different (*P* = 0.045) for kidney and liver with a positive correlation (0.413).

### 3.11. Correlation for Glutathione of Infected and Control Groups

The table (Table 7) provides a correlation analysis for glutathione, and the result shows significant difference (*P* = 0.035) in correlation for serum and kidney with a positive correlation (0.433), no significant different (*P* = 0.42) for serum and liver with positive correlation (0.173), and significant different (*P* = 0.022) for kidney and liver with a positive correlation (0.465).

### 3.12. Kidney Sections of Control and Infected Experimental Wistar Rats (Subacute and Chronic)

In Figure 5, photomicrograph of a kidney section of control in Wistar rat showing intact histology of the glomerulus (G) showing the Bowman's spaces (black arrows) was presented. Both the proximal and distal convoluted tubules were equally visible.

In Figure 6, a photomicrograph of a kidney section of Wistar rats in the 5th day of parasitemia (subacute stage) showing normal glomerulus (G) and slightly degenerated (black arrow) glomeruli. The Bowman's spaces (black arrows) were slightly dilated both the proximal and distal convoluted tubules were equally visible.

In Figure 7, a photomicrograph of a kidney section of Wistar rat 11th day parasitemia (chronic stage) showing normal glomeruli (G) and degenerated (red dashed circle) glomeruli featuring dilated Bowman's capsule (black arrow). Both the proximal (red arrow) and distal convoluted tubules (DCT) were visibly dilated, collapsed, and joined the capsule, thus increased its size.

### 3.13. Liver Sections of Control and Infected Experimental Wistar Rats (Subacute and Chronic)

In Figure 8 is a photomicrograph of liver section of Wistar rat of control group. Normal histology of the liver showing central vein (red-dashed circle), radiating sinusoids (black arrow), and hepatic cords (HC) was presented.

In Figure 9, a photomicrograph of liver section of Wistar rat in the 5th day of parasitemia showing slightly obstructed central veins (red-dashed circles) and with dilated hepatic sinusoids (black arrows).

In Figure 10, a photomicrograph of liver section of Wistar rat in the 11th day of parasitemia (chronic stage) showing completely obstructed and degenerated central veins (red-dashed circles) and with dilated hepatic sinusoids (black arrows).

### 3.14. Spleen Sections of Control and Infected Experimental Wistar Rats (Subacute and Chronic)

In Figure 11, histology of a spleen section from Wistar rat of control group is presenting normal histology of white pulps (dashed circle), patches of splenic cords (black arrows), and radiating splenic sinusoids (red arrows) in the red pulp.

In Figure 12, histology of a section of spleen from Wistar rat in the 5th day of parasitemia (subacute stage) is presenting intermix of normal (black-dashed circle) and necrotic (red-dashed circle) patches of the white pulp.

In Figure 13, histology of spleen section of Wistar rat in the 11th day of parasitemia (chronic stage) showing completely degenerated white pulps (red-dashed-circle) interspersed by red pulp patches of the white pulp.

## 4. Discussion

The first question in the study sought to determine the disease indices of trypanosomiasis. Previous studies have reported an increase in body temperature, a decrease in body weight, and even death if there is no drug intervention. The results of this study follow the same pattern: an increase in body temperature and a decrease in body weight and death, as reported by Balogun et al. [16], Abenga et al. [19], and Mbaya et al. [20]. The increase in body temperature may be a result of contact between the parasite and the defense system of the host. The decrease in weight is due to a loss of appetite by the host during the fight between the host immune system and the parasite for survival.

The hematological indices of the infected and control groups indicate a significant decrease (*P* value = 0.001) in PCV of infected groups (chronic stage 20.46 ± 1.36^bdf^ and subacute stage 27.87 ± 2.21^ab^) to the control groups (chronic stage control 32.57 ± 1.81^f^ and subacute stage control 34.72 ± 0.54^ad^). From the results, the chronic stage has a lower mean PCV than the subacute stage, indicating morbidity of the disease is higher in the chronic stage than the subacute stage. The reduction in PCV is connected with the accelerated destruction of RBC by the immune cells, suppression of the bone marrow response by cytokines, and increased spleen Clarence of infected RBC. However, this agrees with the findings of Omer et al. [12], Maigari and Dabo [9], and Rahul et al. [10]. However, anemia may perhaps be classified as regenerative or nonregenerative according to the bone marrow response; normocytic (normal MCV), macrocytic (amplified MCV), or microcytic (reduced MCV) according to the cell size; and normochromic (normal Hgb), hypochromic (reduced Hgb), or hyperchromic (amplified Hgb) according to the hemoglobin concentrations. Hgb levels in infected groups (chronic stage 6.820.45^bdf^ and subacute stage 9.280.74^ab^) are significantly lower than in the control group (chronic stage 10.870.60^f^ and subacute stage 11.580.18^ad^), *P* value = (0.001). The subacute stage and controls show a normochromic Hgb while the infected chronic stage group shows a hypochromic Hgb, which may be due to the hemolysis of RBC, toxic substances secreted by trypanosome such as neuraminidase and oxidative hemolysis from the product of peroxidation caused by low antioxidant ability of the RBC. The results of the subacute stage and the controls corroborate with the findings of Omer et al. [12], Maigari and Dabo [9], and Rahul et al. [10], while the chronic stage group shows a diverse result, which may be attributed with the morbidity of the disease. A significant decrease *P* value (<0.001) in MCV of the infected group (chronic stage 53.80 ± 1.56^bdf^ and subacute stage 61.44 ± 2.09^b^) to the control group (chronic stage control 66.41 ± 1.92^f^ and subacute stage control 67.86 ± 0.33^d^) was observed, and this indicates a normocytic MCV for the subacute stage group and control groups, while the chronic stage group shows a microcytic MCV. The low MCV that is average red blood cell size, in the chromic stage group, may be due to the morbidity of the disease and iron deficiency, which is likely to be attributed to low feed intake by the animals allocated to the group. Omer et al. [12], Maigari and Dabo [9], and Rahul et al. [10] reported a similar result for MCV in trypanosomiasis. The results for MCH (amount of Hgb per red blood cell) indicate a significant decrease in *P* value (<0.001) in the MCH of the infected group (chronic stage 17.92 ± 0.51^bdf^ and subacute stage 20.47 ± 0.69^b^) to that of the control groups (chronic stage control 22.16 ± 0.64^f^ and subacute stage control 22.64 ± 0.12^d^). RBC has a significantly decrease *P* value (<0.001) in the infected group (chronic stage group 3.78 ± 0.14^bdf^ and subacute stage 4.50 ± 0.21^b^) to the control group (chronic stage control 4.88 ± 0.15^f^ and subacute stage control 5.12 ± 0.09^d^). The mean of chronic stage group for MCH and RBC is significantly lower than the mean of subacute stage and the control groups, this is because morbidity is higher in the chronic stage than subacute stage, and the continuous peroxidative damage to red blood cells can be a key factor. The result of MCHC indicated a decrease (*P* value = 0.747) in MCHC of chronic stage (33.30 ± 0.03), compare to subacute stage (33.31 ± 0.05), subacute stage control (33.31 ± 0.06), and chronic stage control (33.37 ± 0.03). These findings support the findings of Omer et al. [12] and Maigari and Dabo [9] by revealing lower hematological indices. The hematological indices result as suggested by Maigari and Dabo [9] and can continuously be explored as a useful indicator of trypanosomiasis, so it is also suggested from this findings that hematological indices can be used as biomarker of oxidative stress in trypanosomiasis.

Another important finding was the level of antioxidant enzymes in serum, kidney, and liver. Antioxidant defense mechanism functions by inhibiting the initial production of free radicals, neutralizing and oxidizing them into less toxic compounds, inhibiting the secondary production of toxic metabolite or inflammatory mediators, stopping chain generation of secondary oxidants, and reforming the molecular injuries induced by the free radicals [25]. Mammalian red blood cells utilize different antioxidant defenses that work in to cope with free radical generation in the biological system. SOD catalyzes the dismutation of O_2_ to H_2_O_2_. CAT and GSH function to catalyze the degradation of H_2_O_2_ to H_2_O and O_2_.

Serum SOD levels increased significantly (*P* value 0.03) in the infected group (subacute stage 6.240.60 and chronic stage 7.690.80) compared to the control groups (subacute stage 5.210.97 and chronic stage 4.700.44). The variation that occurs between the subacute and chronic stage may be due to the stages of parasite development, which will determine the site of action and localization of the enzyme since the parasite localizes tissue before coming to the peripheral blood and the immunity of the host might play a great role. These is in support with the findings of Yusuf et al. [15] where increase in serum SOD was observed in infected (68.3 ± 5.89) to the control group (65.00 ± 6.97), and Aleksandro et al. [14] also reported an increase in rats infected with *T. evansi*. However, Saleh et al. [8] revealed a significant reduction in the infected *T. evansi* (3.12 ± 0.22) and control (4.62 ± 0.32) group. Similarly, Omer et al. [12] reported a significant reduction in the blood of control (1487.24 ± 78.56) and infected rats (1310.64 ± 178.91), Ogbunugafor et al. [26] reported no significant reduction in serum of rats infected with *T. brucei*. This contradiction might be as a result of the animal model used for the experiment, parasite species and virulence, immunology of the host, and the geographical location, which may interfere with the physiology of the experimental animals. The kidney SOD points out an increase (*P* value = 0.23) with mean value for infected groups (chronic stage 11.06 ± 2.57 and subacute stage 6.63 ± 1.43) to the control groups (chronic stage control 6.02 ± 1.98 and subacute stage control 5.97 ± 1.65). This result is consistent with the findings of Yusuf et al. [15], who found an increase in kidney SOD (37.67 19.67) (24.71 21.96) of infected Wistar rats compared to control Wistar rats, and contradicts the findings of Orhue and Amegor [11], who found a significant decrease in kidney SOD (12.73 1.19; 6.63 1.06; in infected rabbits compared to the control group) in infected rabbits. However, when exposed to oxidative stress, antioxidant enzyme activity increases [27]. The increase in kidney SOD found in this study could be attributed to an increase in oxidant levels caused by trypanosomal infections, which results in mopping up the oxidants to avoid oxidative stress. Furthermore, the kidney functions in blood ultrafiltration; thus, oxidants generated by parasite RBC destruction and cellular respiration tend to be concentrated in the kidney, causing SOD aggregation in the kidney to neutralize the oxidants, and congestion may also occur as a result of glomeruli destruction by toxins and oxidative stress. These can best describe the variation between the subacute stage and chronic stage of infection. The liver SOD levels are significantly lower (*P* value = 0.001) in the infected groups (chronic stage 0.060.00^bdf^ and subacute stage 2.670.14^ab^) than in the control groups (chronic stage 3.180.42^f^ and subacute stage 4.220.44^ad^). The mean SOD of chronic stage is significantly lower than mean of the three groups. This is because the parasite has common SOD in the oxidative stress defense system against free radicals, which assist in elimination of 0_2_ [26]. So also, the distraction of central vein and sinusoid in the liver at the chronic stage leads to necrosis and inflammation, causing damage to the liver after the parasite might have migrated to the peripheral blood for its second phase. This will trigger the recovery of damaged cells in a radical free and antioxidant less environment. This agrees with the finding of Yusuf et al. [15], in which reduction in liver SOD (50 ± 16.67) (54.2 ± 29.17) was observed, and the work of Orhue and Amegor [11] where SOD of liver was also reduced (18.74 ± 1.34) (10.27 ± 0.86).

The serum CAT results are similar to those reported by Saleh et al. [8], who found an increase in CAT (16.99 0.73; 15.87 0.84) in the infected group compared to the control group. Similarly, Yusuf et al. [15] found an increase in serum catalase of infected control Wistar rats (0.62 0.50) (0.44 0.69); Aleksandro et al. [14] found an increase in serum CAT of *T. evansi*-infected Rats. These are in agreement with the result of this study where a significant increase (*P* value = 0.029) with mean value for infected groups (chronic stage 1.90 ± 0.24^df^ and subacute stage 1.58 ± 3.03) to control groups (subacute stage control 0.97 ± 0.13^d^ and chronic stage control 0.98 ± 0.09^d^). Increase in serum catalase may be attributed to the observed increase in serum SOD, which increases the rate of 0_2_ dismutation that directly increases the rate of hydrogen peroxide in the biological system coupled with hydrogen peroxide generated by peroxidation of products, and phagocytosis. Kidney CAT reveals a significant increase (*P* value = 0.016) with mean value for infected groups (chronic stage 15.33 ± 0.56^d^ and subacute stage 13.67 ± 0.68) to control groups (chronic stage control 8.43 ± 1.00 and subacute stage control 7.11 ± 3.55^d^). Liver CAT shows an increase (*P* value = 0.008) with mean value for infected groups (chronic stage 3.16 ± 0.19^df^ and subacute stage 2.56 ± 0.21^a^) to the control groups (chronic stage control 2.08 ± 0.24^f^ and subacute stage control 2.08 ± 0.18^ad^). This supports the findings of Yusuf et al. [15], who found an increase in kidney CAT (1.28 0.96) (1.08 0.27) and liver CAT (1.21 1.08) (0.57 0.34) in infected versus control Wistar rats. This result contradicts the findings of Orhue and Amegor [11] that reported a decrease in kidney CAT (2.01 ± 0.12) (1.07 ± 0.18) and liver CAT (3.45 ± 0.22) (1.14 ± 0.16) of control and infected rabbit. Yusuf et al. [15] reported that under condition of oxidative stress, activities of antioxidant enzymes such as SOD, CAT, and glutathione peroxidase increase, although the parasite lacks CAT in its system and so only the host battle with hydrogen peroxide. Despite the fact that trypanothione [N1,N8-BIS (gluthonyl) spermidine] has been shown to participate not only in oxidant damage to the parasite but also in defense against ribonucleoside metabolism and resistance to antitrypanosomal drugs [28], the host will serve as the alpha in hydrogen peroxide elimination. These may the possible reasons behind the increase in tissue CAT.

The serum GSH from the findings indicates a decrease (*P* value = 0.605) with mean value for infected groups (chronic stage 0.13 ± 0.001 and subacute stage 0.19 ± 0.032), subacute stage control (0.27 ± 0.128), and chronic stage control (0.27 ± 0.109). This result agrees with the findings of Saleh et al. [8] and Rahul et al. [10] that reported a significant reduction in serum GSH (3.88 ± 0.28) (6.85 ± 0.39) and (3.88 ± 0.28) (6.85 ± 0.39) for infected and control groups, and Ismail et al. [29] also reported a decrease in serum GSH. The kidney GSH shows a significant decrease (*P* value = 0.003) with mean value for infected groups (subacute stage 0.70 ± 0.067^a^ and chronic stage 0.43 ± 0.061^c^) to control groups (chronic stage control 0.78 ± 0.156 and subacute stage control 1.02 ± 0.065^ac^). A decrease in liver GSH (*P* value = 0.126) with mean value for infected groups (chronic stage 0.370.050^c^ and subacute stage 0.550.117a) is compared to control groups (subacute stage 0.950.076^ac^ and chronic stage 0.720.130). This contradicts the findings of Yusuf et al. [15], who found an increase in GSH (0.54 0.20) (0.40 0.13) and GSH (0.52 0.26) (0.38 0.10) in the control infected group compared to the uninfected control group. The reduction in serum, kidney, and liver GSH is likely to be caused by the significant increase in serum CAT observed and the activity of trypanothione towards hydrogen peroxide, which will lessen the potential of GSH expression. Although two molecules of GSH are require to complete a reaction to eliminate hydrogen peroxide, this may affect its expression in high amount. In report of oxidative stress in trypanosomiasis, this finding is the first of its kind to correlate antioxidant of different tissue in other to provide a base line for diagnosis of the disease.

The findings on correlation analysis for SOD show a significant (*P* value = 0.036) +ve correlation in serum/liver SOD. This implies that serum and kidney SOD could be more reliable if used as biomarkers of oxidative stress in trypanosome infection. However, the kidney/liver (*P* value = 0.332) and serum/kidney (*P* value = 0.151) SOD show a –ve correlation without statistical significance. Although these results are preliminary, they support the use of serum/liver SOD enzymes for the identification of trypanosome infection. Correlation analysis for CAT shows a significant (*P* value = 0.011) +ve correlation in serum/liver, kidney/liver (*P* value = 0.045), and serum/kidney (*P* value = 0.036). This implies serum/liver, kidney/liver, and serum/kidney can be used if used as biomarkers of oxidative stress in trypanosome infection. Correlation analysis for GSH reveals no statistical significance (*P* value = 0.445), but a positive correlation in serum/liver and serum/kidney (*P* value = 0.853), with kidney/liver showing statistical significance (*P* value = 0.023). This implies that kidney/liver GSH could be more reliable if used as biomarkers of oxidative stress in trypanosome infection. The possible explanation for this result is the level of the enzymes in the serum, kidney, and liver. It can be suggested that CAT could be more reliable as biomarker than SOD and GSH, if used.

High production of reactive oxygen species may result into oxidative stress, ultimately apoptosis or necrosis, and loss of cell function [30]. The kidney of the infected group suffers from subacute to chronic damage, which may be attributed to parasitemia and the level of oxidative stress [31, 32]. The dilation of glomeruli and distil convoluted tubule in the kidney may be as a result of increase in cytokines such as tissue necrotic factor, which causes inflammation [17]. Embolism, thrombosis, and hyperplasia causing glomerulonephritis have been reported to cause damages in trypanosome infection [16, 17]. The liver also showed progressive damage from the subacute to the chronic stage, which could be attributed to parasitemia and oxidative stress levels. These damage in hepatic sinusoids and obstructed central veins may be caused by embolism, thrombosis, and hyperplasia, which may ultimately lead to hypoxia. This might be the reason behind the obstruction of central vein, causing vasculitis and cellular infiltration predominantly by plasma cells. Jake and Wen [13] proposed that MnSOD deficiency exacerbates the loss of mitochondrial function and oxidative phosphorylation capacity and increases myocardial oxidative damage in chagasic cardiomyopathy, which may coincide; this can be used to support the evidence behind the decrease in liver SOD and GSH as part of the reason for the infected groups' liver damage. The spleen also showed shows a progressive damage from the subacute to the chronic, which may also be attributed to increase in dead RBC and WBS concentration and level of oxidative stress. The necrosis observed in the spleen is due to hyperplasia caused by hypercellularity in the spleen, which may be accompanied with vasculitis and cellular infiltration by plasma cells [16, 17]. Jake and Wen [13] conclude with the facts that MnSOD deficiency exacerbates the loss in mitochondrial function and oxidative phosphorylation capacity and enhances the myocardial oxidative damage in chagasic cardiomyopathy, and this may coincide with the destruction of the liver, which is coupled with reduction in liver SOD.

## 5. Conclusion

From the findings of this research, it can be concluded that the disease indices evaluated on infected Wistar rats result in significant decrease in body weight and temperature compared to the control Wistar rats. The second major finding was the erythrocyte indices of infected Wistar rats, and the result shows a significant decrease (*P* value < 0.05) in PCV, Hgb, MCV, MCH, RBC, and MCHC. The study of antioxidant enzymes in infected Wistar rats revealed a significant increase in serum (*P* value = 0.03) and liver SOD (0.001), as well as an increase in kidney SOD (*P* value = 0.23). The CAT in serum (*P* value = 0.011), liver (*P* value = 0.016), and kidney (*P* value = 0.008) increased and are statistically significant. GSH levels are significantly higher in the kidney and liver (*P* value 0.05), but lower in the serum (*P* value = 0.605). The results of histology revealed that tissue distortion progressed with infection stage.

## Figures and Tables

**Figure 1:** Mean body weight of experimental Wistar rats infected with *T. brucei brucei* under subacute and chronic stages.

**Figure 2:** Mean body temperature of experimental Wistar rats infected with *T. brucei brucei* under subacute and chronic stages.

**Figure 3:** Mean parasitemia of experimental Wistar rats infected with *T. brucei brucei* under subacute and chronic stages.

**Figure 4:** Percentage survival of experimental Wistar rats infected with *T. brucei brucei* under subacute and chronic stages.

**Figure 5:** Photomicrograph of a kidney section of control Wistar rat.

**Figure 6:** A photomicrograph of a kidney section of subacute stage Wistar rat.

**Figure 7:** A photomicrograph of a kidney section of chronic stage Wistar rat.

**Figure 8:** Photomicrograph of a liver section of control Wistar rats.

**Figure 9:** A photomicrograph of a liver section of subacute stage Wistar rat.

**Figure 10:** A photomicrograph of a liver section of chronic stage Wistar rat.

**Figure 11:** Photomicrograph of a spleen section of control Wistar rats.

**Figure 12:** Photomicrograph of a spleen section of subacute stage Wistar rats.

**Figure 13:** Photomicrograph of a spleen section of chronic stage Wistar rats.

**Table 1:** Mean ± standard error of hematological indices of experimental Wistar rats infected with *T. brucei brucei* under subacute and chronic stages.

	5th day Prst SAC (*n* = 6)	Control 5th day Prst CSAC (*n* = 6)	11th day Prst CR (*n* = 6)	Control 11th day Prst CCR (*n* = 6)	*P* value
PCV (%)	27.87 ± 2.21^ab^	34.72 ± 0.54^ad^	20.46 ± 1.36^bdf^	32.57 ± 1.81^f^	<0.001
Hgb (g/dL)	9.28 ± 0.74^ab^	11.58 ± 0.18^ad^	6.82 ± 0.45^bdf^	10.87 ± 0.60^f^	<0.001
MCHC (g/dL)	33.31 ± 0.05	33.31 ± 0.06	33.30 ± 0.03	33.37 ± 0.03	0.747
MCV (fl)	61.44 ± 2.09^b^	67.86 ± 0.33^d^	53.80 ± 1.56^bdf^	66.41 ± 1.92^f^	<0.001
MCH (pg)	20.47 ± 0.69^b^	22.64 ± 0.12^d^	17.92 ± 0.51^bdf^	22.16 ± 0.64^f^	<0.001
RBC (10^6^/*μ*L)	4.50 ± 0.21^b^	5.12 ± 0.09^d^	3.78 ± 0.14^bdf^	4.88 ± 0.15^f^	<0.001

Means with similar superscript along the column show significant different when *P* < 0.05. Keys: Prst: parasitemia; SAC: subacute stage; CSAC: control subacute stage; CR: chronic stage; CCR: control chronic stage; PCV: pack cell volume; Hgb: hemoglobin; *n*: number of rats; MCV: mean corpuscular volume; MCH: mean corpuscular hemoglobin; RBC: red blood cell; MCHC: mean corpuscular hemoglobin concentration.

**Table 2:** Superoxide activity of experimental Wistar rats infected with *T. brucei brucei* under subacute and chronic stages.

	5th day Prst SAC (*n* = 5)	Control 5th day Prst CSAC (*n* = 5)	11th day Prst CR (*n* = 5)	Control 11th day Prst CCR (*n* = 5)	*P* value
Serum (U/mL)	6.74 ± 0.60	5.21 ± 0.97	7.69 ± 0.80	4.70 ± 0.44	0.033
Kidney (U/g)	6.63 ± 1.43	5.97 ± 1.65	11.06 ± 2.57	6.02 ± 1.98	0.23
Liver (U/g)	2.67 ± 0.14^ab^	4.22 ± 0.44^ad^	0.06 ± 0.00^bdf^	3.18 ± 0.42^f^	<0.001

Means with similar superscript along the column shows significant different when *P* < 0.05. Keys: Prst: parasitemia; SAC: subacute stage; CSAC: control subacute stage; CR: chronic stage; CCR: control chronic stage; *n*: number of rats.

**Table 3:** Mean ± standard error of catalase of experimental Wistar rats infected with *T. brucei brucei* under subacute and chronic stages.

	5th day Prst SAC (*n* = 5)	Control 5th day Prst CSAC (*n* = 5)	11th day Prst CR (*n* = 5)	Control 11th day Prst CCR (*n* = 5)	*P* value
Serum (U/mL)	1.58 ± 3.03	0.97 ± 0.13^d^	1.90 ± 0.24^df^	0.98 ± 0.09^d^	0.011
Kidney (U/g prot)	13.67 ± 0.68	7.11 ± 3.55^d^	15.33 ± 0.56^d^	8.43 ± 1.00	0.016
Liver (U/g prot)	2.56 ± 0.21^a^	2.08 ± 0.18^ad^	3.16 ± 0.19^df^	2.08 ± 0.24	0.008

Means with similar superscript along the column shows significant different when *P* < 0.05. Keys: Prst: parasitemia; SAC: subacute stage; CSAC: control subacute stage; CR: chronic stage; CCR: control chronic stage; *n*: number of rats.

**Table 4:** Mean ± standard error of reduced glutathione of experimental Wistar rats infected with *T. brucei brucei* under subacute and chronic stages.

	5th day Prst SAC (*n* = 5)	Control 5th day Prst CSAC (*n* = 5)	11th day Prst CR (*n* = 5)	Control 11th day Prst CCR (*n* = 5)	*P* value
Serum (g/L)	0.19 ± 0.032	0.27 ± 0.128	0.13 ± 0.001	0.27 ± 0.109	0.605
Kidney (mg/g prot) 0.70 ± 0.067^a^	1.02 ± 0.065^ac^	0.43 ± 0.061^c^	0.78 ± 0.156	0.003	
Liver (mg/g prot)	0.55 ± 0.117^a^	0.95 ± 0.076^ac^	0.37 ± 0.050^c^	0.72 ± 0.130	0.003

Means with similar superscript along the column shows significant different when *P* < 0.05. Keys: Prst: parasitemia; SAC: subacute stage; CSAC: control subacute stage; CR: chronic stage; CCR: control chronic stage; *n*: number of rats.

**Table 5:** Correlation for superoxide dismutase of experimental animals.

Variables	Serum SOD (U/mL)	
	*r*	*P* value
Kidney SOD (U/g) (*N* = 24)	-0.302	0.151
Liver SOD (U/g) (*N* = 24)	0.431^∗^	0.036
	Kidney SOD (U/g)	
Liver SOD (U/g) (*N* = 24)	-0.207	0.332

^∗^Correlation is significant at the 0.05 level (2-tailed).

**Table 6:** Correlation for catalase of experimental animals.

Variables	Serum CAT (U/mL)	
	*r*	*P* value
Kidney CAT (U/g) (*N* = 24)	0.430^∗^	0.036
Liver CAT (U/g) (*N* = 24)	0.511^∗^	0.011

	Kidney CAT (U/g)	
Liver CAT (U/g) (*N* = 24)	0.413^∗^	0.045

^∗^Correlation is significant at the 0.05 level (2-tailed).

**Table 7:** Correlation for reduced glutathione of experimental animals.

Variables	Serum GSH (g/L)	
	*r*	*P* value
Kidney GSH (mg/g) (*N* = 24)	-0.046^∗^	0.853
Liver GSH (mg/g) (*N* = 24)	0.164	0.445
	Kidney GSH (mg/g)	
Liver GSH (mg/g) (*N* = 24)	0.461^∗^	0.023

^∗^Correlation is significant at the 0.05 level (2-tailed).

## Data Availability

The numeric and histological data used to support the findings of this study are included within the article.
